The article "A Novel and Effective Brain Tumor Classification Model Using Deep Feature Fusion and Famous Machine Learning Classifiers" was published in 2022. Journal: Comput Intell Neurosci.

# A Novel and Effective Brain Tumor Classification Model Using Deep Feature Fusion and Famous Machine Learning Classifiers

**DOI:** 10.1155/2022/7897669

**Published:** 2022-03-26

**Authors:** Hareem Kibriya, Rashid Amin, Asma Hassan Alshehri, Momina Masood, Sultan S. Alshamrani, Abdullah Alshehri

**Affiliations:** ^1^Department of Computer Science, University of Engineering and Technology, Taxila, Pakistan; ^2^Durma College of Science and Humanities Shaqra University, Shaqra 11961, Saudi Arabia; ^3^Department of Information Technology, College of Computer and Information Technology, Taif University, P.O. Box 11099, Taif 21944, Saudi Arabia; ^4^Department of Information Technology, Al Baha University, Al Bahah, Saudi Arabia

## Abstract

Brain tumors are difficult to treat and cause substantial fatalities worldwide. Medical professionals visually analyze the images and mark out the tumor regions to identify brain tumors, which is time-consuming and prone to error. Researchers have proposed automated methods in recent years to detect brain tumors early. These approaches, however, encounter difficulties due to their low accuracy and large false-positive values. An efficient tumor identification and classification approach is required to extract robust features and perform accurate disease classification. This paper proposes a novel multiclass brain tumor classification method based on deep feature fusion. The MR images are preprocessed using min-max normalization, and then extensive data augmentation is applied to MR images to overcome the lack of data problem. The deep CNN features obtained from transfer learned architectures such as AlexNet, GoogLeNet, and ResNet18 are fused to build a single feature vector and then loaded into Support Vector Machine (SVM) and K-nearest neighbor (KNN) to predict the final output. The novel feature vector contains more information than the independent vectors, boosting the proposed method's classification performance. The proposed framework is trained and evaluated on 15,320 Magnetic Resonance Images (MRIs). The study shows that the fused feature vector performs better than the individual vectors. Moreover, the proposed technique performed better than the existing systems and achieved accuracy of 99.7%; hence, it can be used in clinical setup to classify brain tumors from MRIs.

## 1. Introduction

Brain tumors are one of the most dangerous types of brain diseases that can develop due to abnormal cell growth inside the skull. Brain tumors can be categorized into two types: primary tumors and secondary tumors. Primary brain tumors account for 70% of all tumors and spread only in the brain, whereas secondary brain tumors form in other organs such as the breast, kidney, and lung before migrating to the brain. According to a study by NBTF, in US alone, around 29,000 cases of primary brain tumor are diagnosed each year, resulting in the death of 13,000 people [1]. Similarly, in the United Kingdom, about 42,000 people with primary brain tumors die each year. Glioma, Meningioma, and Pituitary tumors are the most prevalent brain tumors. Glioma tumor is caused by unusual growth in Glial cells that constitute 80% of the brain. Among all primary tumors, it has the highest fatality rate. Meningioma tumors develop in the brain's protective membrane, the meninges spinal cord. In contrast, the pituitary tumor develops in the pituitary gland. This gland produces various necessary hormones. Although the pituitary tumor is benign, it can cause hormonal deficiencies and irreparable damage to vision [2]. Hence, an early and accurate diagnosis of brain tumors is necessary to protect patients from damaging effects [3]. Depending on their objective, brain tumors can be diagnosed using various medical imaging technologies. Ultrasonography (US), magnetic resonance imaging (MRI), and computed tomography (CT) are three of the widely used techniques [4]. The most prevalent noninvasive imaging technology is magnetic resonance imaging (MRI), which does not emit any harmful ionizing radiation during the examination like X-rays. Furthermore, it generates clear images of soft tissues and can acquire modalities like FLAIR, T1, and T2, using a variety of parameters [5].

The article "A Novel and Effective Brain Tumor Classification Model Using Deep Feature Fusion and Famous Machine Learning Classifiers" was published in 2022. Journal: Comput Intell Neurosci.

Proper identification of tumor type is a difficult task as the tumors usually vary in shape, intensity, size, and location. Usually, the medical professionals visually inspect the images and meticulously mark out the tumor regions in the images. Because of the surrounding healthy tissues, tumor borders are frequently blurred. As a result, the manual identification process via optical inspection is time-consuming and can cause misinterpretation of the tumor. Furthermore, manual tumor detection relies heavily on the radiologist's experience [6]. It should also be mentioned that the human eye cannot distinguish between distinct shades of grey shown in MRI scans. Other prominent reasons for tumor misinterpretation include fatigued radiologists or noisy MRIs caused by variations in imaging devices. Thus, automated systems are appropriate when radiologists want to visually evaluate the depth of the tumor or identify the type of tumor to reduce the likelihood of biopsy [7, 8]. Various researchers have proposed CAD-based brain tumor detection methods. However, the limitation of traditional ML-based algorithms is that they use a hand-crafted feature extraction strategy. The features are extracted from training images before classification [9].

The article "A Novel and Effective Brain Tumor Classification Model Using Deep Feature Fusion and Famous Machine Learning Classifiers" was published in 2022. Journal: Comput Intell Neurosci.

Brain tumor classification techniques can be divided into machine learning- (ML-) based methods and deep learning- (DL-) based methods. The ML-based systems employ handcrafted feature extraction and manual segmentation before classification that is time-consuming and error-prone. These methods typically require the assistance of an expert with extensive experience to discover optimal feature extraction and segmentation algorithms for proper tumor identification. As a result, when working with larger databases, the performance of these systems is prone to errors [10]. Meanwhile, DL-based algorithms perform these steps automatically and have proven incredibly useful in various applications, including medical image analysis. One of the most prominent DL models, i.e., convolutional neural network (CNN), is widely employed because of its robust performance and weight-sharing nature. It can extract low- level and high-level features from training data automatically. Hence, these techniques have drawn the interest of scientists and researchers [11, 12].

This paper is a continuation of research presented in Kibriya et al. [9] that compares the performance of two transfer learning architectures such as ResNet18 and GoogLeNet to classify brain tumors from MRI images. The deep features were classified using end-to-end CNN models as well as ECOC based SVM. This paper proposes an automated method based on the fusion of deep features obtained via three well-known CNNs, AlexNet, ResNet18, and GoogLeNet, for brain tumor identification and classification. Feature fusion is a method that combines multiple low and high-level features into a single feature vector, thus increasing the discrimination performance of model by eliminating the need of utilizing feature vector from a single model. The motivation behind using a feature fusion-based technique is to produce informative and discriminative features from MRIs, which are critical for accurate tumor classification. To demonstrate the efficacy of the suggested method, we used multiple quantitative measures to assess our model on a well-known brain tumor dataset [13]. The primary contributions of the proposed system are as follows:

- We designed a completely automated hybrid system that uses both (a) transfer learned CNN models for deep feature extraction and (b) ML classifiers for effective classification of the type of brain tumors.
- The proposed method consists of five core steps such as (a) image intensity normalization, (b) extensive dataset augmentation, (c) feature extraction via multiple CNNs, that is, AlexNet, ResNet18, and GoogLeNet, (d) fusion of deep features vector that achieves cutting-edge performance for classifying brain tumors from MR images, and (e) tumor type classification via SVM and KNN.
- The concatenation of deep features in a single vector enhances the discriminating power. It enables effective tumor classification under various challenges such as complex background, fuzzy tumor boundaries, varying tumor location, and other problems in MRI artifacts.
- The obtained results show the robustness of the proposed approach compared to existing systems.

The article "A Novel and Effective Brain Tumor Classification Model Using Deep Feature Fusion and Famous Machine Learning Classifiers" was published in 2022. Journal: Comput Intell Neurosci.

The paper is arranged as follows.  Section 2 analyzes related studies.  Section 3 describes the proposed method.  Section 4 and Section 5 are dedicated to experiments and results, respectively. The proposed work is concluded in Section 6.

## 2. Literature Review

Early tumor identification and classification of brain tumors are necessary for the effective treatment of a patient. Experts can now provide better treatment to patients via automated healthcare systems because of remarkable technology improvements. The researchers have proposed studies employing ML and DL based algorithms to solve medical image diagnosis problems [14]. One of the most famous DL models is CNN, which has achieved groundbreaking results in different fields, including image processing. CNN-based systems can efficiently diagnose brain tumors and assist healthcare providers in determining treatment decisions for patients. According to the statistics of 2016, more than 200 DL-based researches on medical images were proposed, and 190 of those employed the CNNs [11]. Some of the very popular CNNs such as AlexNet [15], VGG [16], and GoogLeNet [17] are currently being used in medical image classification tasks. This section discusses the recent studies for brain tumor classification in detail.

Mzoughi et al. [18] demonstrated 3D CNN architecture for glioma brain tumor classification into low-grade gliomas (LGG) and high-grade gliomas (HGG) utilizing the entire volumetric T1-Gado MRI sequence from Brats 2018 dataset. Using small kernels, the architecture combined local and global contextual information with lower weights, based on a 3D convolutional layer and a deep network. The system achieved 96.49% accuracy. Maqsood et al. [19] suggested a brain tumor detection method employing edge detection and U-NET model. The tumor segmentation framework enhances image contrast and performs edge detection fuzzy logic. The features are extracted from decaying subband images and then classified using the U-NET architecture, which detects the presence of meningioma in brain images. Togacar et al. [20] developed BrainMRNet using attention modules and the hypercolumn method. Initially, the images were preprocessed before being sent to the attention modules. Attention modules determine the key regions of an image and send the image to convolutional layers. Hypercolumn is one of the important techniques used by the BrainMRNet model in the convolutional layers. The features extracted from each layer are maintained by the array structure in the final layer using this technique. The system achieved an accuracy of 96.05%. The authors in Khawaldeh et al. [21] suggested a CNN model to detect brain tumors and Glioma tumors by improving pretrained architecture and achieving 91% overall accuracy. Despite the tremendous amount of work in this field, developing a good and practical technique for classifying brain MR images still requires additional research. The main limitation of the research in [18–21] is that they only perform binary classification of brain tumors and disregard multiclass classification, requiring additional analysis to determine the kind of tumor.

The article "A Novel and Effective Brain Tumor Classification Model Using Deep Feature Fusion and Famous Machine Learning Classifiers" was published in 2022. Journal: Comput Intell Neurosci.

Several recent researches employing transfer learning-based methods to detect brain tumors have been proposed. For example, the authors in Sajjad et al. [22] demonstrated a multimodal tumor classification system based on CNN. They initially segmented the MR images using Input Cascade CNN and classified them using a fine-tuned VGG-19 with 94.5% accuracy. However, the framework is computationally inefficient as it performs segmentation and classification via CNNs. Ari et al. [23] fused deep features obtained from AlexNet and VGG16. The fused feature vector was then classified via Extreme Learning Machine (ELM). The study was conducted on MRI images from publicly available Figshare, Rider, and REMBRANDT datasets. The system achieved 96.6% accuracy. Noreen et al. [24] extracted deep features using VGG16, VGG19, and AlexNet and classified the features via ensemble classifiers. The system achieved the highest accuracy of 94.3%. Swati et al. [25] classified brain tumor MRI images using fine-tuned AlexNet and VGG with an accuracy of 94.8%. The authors in Saxena et al. [26] employed ResNet, Inception-V3, and VGG-16 and achieved the highest accuracy of 95% via ResNet. However, the techniques obtained a low overall performance and need to be tested before real-time deployment.

The authors in Abiwinanda et al. [27], on the other hand, suggested five CNN designs to classify brain tumors and obtained the highest validation accuracy of 84.1%. It may be noted that very simplistic CNNs cannot extract deep high-level features, resulting in poor overall accuracy. Alanazi et al. [28] presented a brain tumor classification framework employing novel 22 layered CNN architectures and achieved the highest accuracy of 96.8%. However, the proposed technique is trained and evaluated on limited imaging samples. Khan et al. [29] proposed a Hierarchical Deep Learning-Based Brain Tumor classification method. The study was conducted on MRI images from Kaggle dataset and achieved 92.13% classification accuracy. However, the system needs to be tested before deploying for clinical setup for brain tumor classification due to low overall accuracy. Anaraki et al. [30] employed the Genetic Algorithms (GA) to find an optimal CNN architecture with lesser computation cost for the classification of brain tumors. They obtained 94.2% accuracy to classify Glioma, Meningioma, and Pituitary tumors from MRI images. However, GA could not find optimal CNN architecture, thus resulting in poor overall accuracy. The authors in Raja [31] employed Bayesian fuzzy clustering (BFC) technique for image segmentation, nonlocal mean filter for image denoising and scattering transform, information-theoretic measurements, and wavelet packet Tsallis entropy for feature extraction and a hybrid DAE strategy for brain tumor classification. However, this technique takes a long time to compute and is computationally inefficient. Afshar et al. [32] used Capsule Networks to identify and classify brain lesions with 90.89%. It should be noted that CapsNets are particularly sensitive to image backgrounds and perform better when segmented images are used to train the model. As a result, the architecture is complicated.

The article "A Novel and Effective Brain Tumor Classification Model Using Deep Feature Fusion and Famous Machine Learning Classifiers" was published in 2022. Journal: Comput Intell Neurosci.

## 3. Proposed Methodology

This paper proposes a novel MRI-based brain tumor identification and classification method employing a fusion of deep CNN features. The workflow diagram is presented in Figure 1. The MRI images are normalized and augmented before being fed into three separate CNN models for feature extraction. The obtained deep feature vectors are fused in a single feature vector and classified via SVM and KNN. The proposed method is robust and efficient and can be utilized to accurately classify different types of brain tumors such as Pituitary, Glioma, and Meningioma.

### 3.1. Data Preprocessing

MRI images from the dataset are initially preprocessed by applying min-max normalization, as explained in equation (1). The intensity values in an image are scaled between [0, 1] by applying the normalization technique. This normalization technique transforms the minimum value of the feature to 0 and the maximum value to 1.

(1) $$\begin{array}{c} f\left(x,y\right)=\frac{f\left(x,y\right)-Z_{\min}}{Z_{\max}-Z_{\min}}, \end{array}$$

where *f* denotes the brain image, *x* and *y* are the pixel's location in an image, the minimum pixel value is indicated by *Z*_min_, and the maximum pixel value by *Z*_max_Figure 2 shows the result of the min-max normalization technique. These images are then rescaled according to the input layer size of the CNNs. The preprocessing steps facilitate network training by speeding up the learning process and solving memory problems.

The article "A Novel and Effective Brain Tumor Classification Model Using Deep Feature Fusion and Famous Machine Learning Classifiers" was published in 2022. Journal: Comput Intell Neurosci.

### 3.2. Image Augmentation

The dataset utilized in this study has a limited number of MRI samples; hence, the preprocessed images are artificially increased by using the various augmentation techniques described as shown in Figure 3. Usually the models tend to be biased towards labelling the new instances as majority class types due to uneven class distribution; hence, this problem can be reduced artificially augmenting the dataset. The images are augmented by applying left/right mirroring, adding salt and pepper noise using density (d) of 0.003, flipping the image around the *x*-axis, and applying 45-degree rotation with bilinear interpolation, in which the output value of the pixel is a weighted average of pixels in the nearest 2-by-2 neighborhood. Dataset augmentation techniques increased the MRI images from 3064 to 15,320 images as shown in Table 1.

### 3.3. Deep Feature Extraction

#### 3.3.1. Convolutional Neural Network

The robust performance of CNNs has increased its popularity among academics and encouraged them to solve previously thought-to-be-impossible issues. In recent years, researchers have built many CNN architectures to address diverse challenges in various disciplines, including medical image identification [33]. CNN is composed of numerous layers stacked on top of one another. CNN's architecture consists of two main parts: (i) feature extraction module employing convolutional layers for learning the features, and pooling layers for downsizing the image dimensions, and (ii) classification module comprising a fully connected (FC) layer for classifying an image [8]. The general architecture of the CNN is illustrated in Figure 4.

#### 3.3.2. Transfer Learning

The CNNs generally perform better on larger datasets than the smaller ones. Training CNN models from scratch requires a lot of resources. Hence, transfer learning is used in situations where it is impossible to build a big training dataset or custom CNN architecture.  Figure 5 demonstrates the concept of transfer learning. A model that has already been trained on bigger datasets such as ImageNet [15] can be used as a feature extractor on a smaller dataset assignment. Transfer learning is being implemented in various fields, including medical image diagnosis and X-ray screening of baggage [34]. This technique decreases the long network training time required for building custom deep learning models and the requirement for a big dataset.

The article "A Novel and Effective Brain Tumor Classification Model Using Deep Feature Fusion and Famous Machine Learning Classifiers" was published in 2022. Journal: Comput Intell Neurosci.

In this study, we employed CNN architectures, namely, AlexNet [15], GoogLeNet [17], and ResNet18 [35], as deep feature extractors since the CNNs are capable of collecting significant features without any human supervision. Furthermore, because the Figshare dataset is not particularly large, we adopt a strategy based on transfer learning to develop our feature vector. It may be noted that training a deep learning model from scratch requires numerous computer resources; thus, we use transfer learned models to aid in learning target domains using source domains and learning tasks [35, 36]. In the proposed study, we employed a transfer learning strategy by modifying the last three layers of the CNNs (i.e., FC, Softmax and Classification) according to our target domain.  Figure 6 shows the general architectures of (a) AlexNet, (b) ResNet, and (c) GoogLeNet. AlexNet was proposed by Alex Keizhevsky that is composed of 8 learnable layers, out of which 5 are Convolution Layers (CLs), and 3 are Fully Connected (FC) layers [15]. Due to its lightweight nature and robust performance, researchers widely use the model for classification tasks. GoogLeNet is a variant of the Inception network developed by researchers at Google. The CNN contains 9 inception modules and is 22 layers deep. The architecture is efficient as it retains the spatial information in an image even after image reduction [17]. The ResNet18 architecture has 18 layers, including 17 CLs, an FC layer, and an additional softmax layer for classification. The CLs use a 3 × 3 sized kernel. The ResNets use shortcut connections that skip one or more layers, thus resulting in a lower training loss, whereas their outputs are added to the outputs of stacked layers; hence, it does not increase the computational complexity. The shortcut connections of ResNet18 skip two layers [35].  Table 2 shows the input size, depth, and parameters of all three CNN architectures used in this study. The input size refers to the size required for an input image. The depth of architecture represents the largest number of sequential CLs or FC layers from the first layer to the classification layer. The parameter shows the total amount of learnable parameters in the entire network.

### 3.4. Fusion of Deep CNN Features

The success of ML classifier is heavily reliant on an input feature vector; thus, developing an algorithm to generate informative and discriminative features from MRIs is crucial for accurate tumor classification. In this phase, we fuse the deep features obtained from the transfer learned CNNs in the previous phase. Feature fusion is a technique that merges numerous features from several different models into a single feature vector, thus avoiding the need to utilize a single feature vector obtained from a model with low overall performance. This integration of features will likely improve classification results as the new feature vector contains more information about the MR images than a single vector [8]. The deep CNN features obtained from two homogenous architectures have identical feature spaces. As a result, the fusion of these features may contain repetitive feature space, thus lacking diversity. Hence, we used heterogeneous CNN architectures with varying architectural design and depth to extract diverse low level and high level features from MR images. The novel fused feature vector contains more information than the independent feature vectors.  Figure 7 depicts the feature fusion procedure employed in the proposed study. Each independent feature vector has three feature spaces according to the number of classes in the dataset; hence, the fused feature vector consists of 9 features.

The article "A Novel and Effective Brain Tumor Classification Model Using Deep Feature Fusion and Famous Machine Learning Classifiers" was published in 2022. Journal: Comput Intell Neurosci.

### 3.5. Classification

In this phase, the novel feature vector is supplied to well-known classifiers such as SVM and KNN. SVM is a supervised learning method belonging to generalized linear classifiers that maximize the margin between the hyperplane and the dataset to boost accuracy and avoid overfitting [37]. The classifier was proposed by Vladimir Wapnik and his team in 1992 [38, 39], whereas KNN was developed by Thomas Cover and has been used successfully for regression and classification tasks in a variety of fields. Since the early 1970s, it has been employed in various statistical applications. It is a supervised learning model that computes the distance between a test sample and a set of (*k*) training samples. The classifier assigns the test sample to the majority category label of its *k* nearest training samples [40]. Both classifiers are frequently utilized in handwriting recognition, medical image problems, etc., due to their robust performance.

## 4. Proposed Method Results

### 4.1. Dataset

The dataset used in this study was published online in 2017 by Jun Cheng. It consists of T1-weighted MRI images of Glioma, Meningioma, and Pituitary tumors taken at three planes, i.e., Coronal, Sagittal, and Axial. The images in the dataset are sized 512 × 512, whereas the size of each pixel is 49 mm × 49 mm. [13]. A detailed description of the dataset in terms of tumor type and no. of plane-wise images with respect to patients is presented in Table 3, whereas Figure 8 displays normalized MRI images from the dataset at different planes.

Figure 9 illustrates the exploratory data analysis to understand the dataset class distribution. The pie chart shows that Glioma samples compose 46% of the entire dataset. Meningioma and Pituitary images account for only 23% and 30% of the overall dataset, respectively. The chart indicates class imbalance issues; hence, in such conditions, Recall, F1-Score, and Precision are more appropriate metrics compared to accuracy.

The article "A Novel and Effective Brain Tumor Classification Model Using Deep Feature Fusion and Famous Machine Learning Classifiers" was published in 2022. Journal: Comput Intell Neurosci.

### 4.2. Experimental Settings

This study employed transfer learning CNNs such as ResNet18, AlexNet, and GoogLeNet as deep feature extractors. For classification, the deep features were fused and supplied to SVM and KNN. All the experiments are performed on an Intel Core i5 processor with an 8 GB RAM using Matlab R2021a. The hyperparameters of the CNN and the values are shown in Table 4.

We trained the CNNs using 30 epochs. This is an epoch when an entire dataset is passed forward and backward through the architecture only once. The epoch is too large to process all at once, so it is usually broken into smaller batches. The total number of training examples in a single batch (or mini-batch) is referred to as a batch size/mini-batch size (such as 10 in our case) [41]. The CNNs in the proposed frameworks are trained on a 1*e* − 4 learning rate. The learning rate determines how quickly an algorithm learns the values of a parameter estimate. It may be noted that higher learning rates frequently result in a suboptimal set of weights [42]. Moreover, we trained the CNNs using stochastic gradient descent momentum (SGDM) optimizer. The SGD optimizes the network parameters to achieve optimal loss function by taking incremental steps towards negative gradient at each iteration. SGD can oscillate along the steepest descent path to the best solution. One method for reducing this oscillation is to include a momentum term in the parameter update [43], as shown in the following equation:

(2) $$\begin{array}{c} \theta_{i+1}=\theta_{i}-\propto \nabla L\left(\theta_{i}\right)+\gamma \left(\theta_{e}-\theta_{i+1}\right), \end{array}$$

where *i* denotes the iteration number, *a* represents learning rate, *θ* is the parameter vector, *L*(*θ*) is the loss function, and *γ* determines the contribution of the previous gradient step to the current iteration in the SGDM algorithm.

### 4.3. Evaluation Metrics

When designing automated systems, evaluating the model's performance is vital because the main purpose of such a model is to forecast unanticipated data reliably; hence, analyzing the training and validation test set reveals the generalization ability of the framework. Usually, a classification model is assessed using a confusion matrix, a simple cross-tabulation of actual and expected observations for each class. Various classification measures based on the confusion matrix, such as accuracy, precision, recall, and *f*1-score, are used as a benchmark to assess the model's performance. The classification accuracy is a popular metric to summarize the model's overall performance. The *f*1-score, on the other hand, combines precision and recall into a single statistic that contains both features. The recall is calculated in equation (3), Precision in equation (4), Accuracy in equation (5), and *F*1-Score in equation (6).

(3) $$\begin{array}{c} \text{Recall}=\frac{\text{TP}}{\text{FN}+\text{TP}}, \end{array}$$

(4) $$\begin{array}{c} \text{Precision }=\frac{\text{TP}}{\text{FP}+\text{TP}}, \end{array}$$

(5) $$\begin{array}{c} \text{Accuracy }=\frac{\text{TN}+\text{TP}}{\text{TP}+\text{FN}+\text{TN}+\text{FP}}, \end{array}$$

(6) $$\begin{array}{c} \text{F}1-\text{Score}=\frac{\text{TP}}{\text{TP}}+\frac{1}{2}\left(\text{FP}+\text{FN}\right), \end{array}$$

where TP = True Positives, TN = True Negatives, FP = False Positives, and FN = False Negatives.

The article "A Novel and Effective Brain Tumor Classification Model Using Deep Feature Fusion and Famous Machine Learning Classifiers" was published in 2022. Journal: Comput Intell Neurosci.

### 4.4. Proposed Method Results

This section discusses the proposed method results.  Table 5 compares the accuracy values obtained via independent CNN feature vectors and novel fused feature vectors. The feature vectors from independent CNN architectures such as ResNet18 and AlexNet achieved the maximum accuracy of 98%, while GoogLeNet produced an accuracy of 97.6%. On the other hand, the fused feature vector obtained an accuracy of 99.7% and outperformed the independent feature vectors.

The performance of our proposed technique is also evaluated using other metrics such as F1-Score, recall, and precision, as shown in Figure 10. The classifiers achieved precision, recall, and *F*1-Score of 0.99, 0.1, and 0.99, respectively. These metrics indicate our proposed method's robustness despite the dataset's class imbalance due to a fused feature vector with more robust and discriminative features than an independent feature vector.  Table 6 shows metrics such as Recall, Precision, and *F*1-Score obtained from the confusion matrix class-wise.

Figure 11(a) shows the confusion matrix obtained from SVM. The *X*-axis of the matrix represents the predicted class, while the *Y*-axis represents the true class. The matrix indicates that SVM correctly classified 2132 Glioma samples, 1051 Meningioma samples, and 1393 Pituitary samples. The confusion matrix obtained on the fused feature vector via KNN is shown in Figure 11(b). The matrix illustrates that KNN correctly identified 2130 Glioma samples, 1052 Meningioma samples, and 1393 Pituitary samples. Both classifiers obtained an accuracy of 99.7%.

Figure 12 shows Receiver Operating Curves (ROC) for all three classes: Glioma, Meningioma, and Pituitary. ROC analysis was originally developed during World War II to analyze noise in the radar signals [44]. The use of ROC curves for assessing the performance of medical diagnostic systems has grown in popularity over the last few decades. The curve indicates the trade-off between specificity and sensitivity. It is more efficient when the curve is closer to the upper left corner. One of the best properties of ROC is that the accuracy indices generated from the analysis are not influenced by fluctuations caused by arbitrarily chosen decision criteria or cut-offs [45]. The area under the ROC curve determines the discriminative capacity showing how efficiently it performs in a certain scenario [46]. An excellent model has an AUC close to one, indicating a high level of separability between the classes.

The article "A Novel and Effective Brain Tumor Classification Model Using Deep Feature Fusion and Famous Machine Learning Classifiers" was published in 2022. Journal: Comput Intell Neurosci.

## 5. Result Comparison with State-of-the-Art Techniques

Recent advancements in medical image analysis tools have provided health practitioners more convenience with detecting diseases at an early stage. Such advancements are assisting them in various fields of medicine, including disease identification, therapy, and quick decision-making for clinical applications. Every day, hospitals generate a large amount of medical data. Medical informatics research assists doctors and scientists in their search for the best solutions for making good use of these ever-increasing volumes of data [47, 48].

Early detection and appropriate treatment options are essential to treat brain tumor illnesses effectively. Those treatment options are determined by the stage of tumor, type, and grade at the diagnosis time. The conventional identification systems employs basic ML-oriented algorithms that extract limited features [7, 49]. This paper presents a novel feature fusion-based strategy to classify brain tumors from MR images accurately.

Table 7 gives a comprehensive comparison of our proposed tumor detection and classification algorithms with the existing methodologies using accuracy as a metric. Afshar et al. [32] classified brain tumors with 90.8% using a CapsNet architecture. However, CapsNet architectures are extremely sensitive to image background, severely impacting the performance. Furthermore, they gave tumor boundaries extra input for improved results, necessitating manual tumor localization prior to classification. Anaraki et al. [30] employed GA to determine optimal CNN design and achieved an accuracy of 94.2%. However, GA was unable to find best CNN for brain tumor diagnosis, thus resulting in low overall accuracy. Kang et al. [8] fused deep features from DenseNet169, Inception-v3, and ResNeXt50 to classify brain tumors. The system obtained a high accuracy of 98.5%. Ari et al. [23] fused deep features obtained from AlexNet and VGG16, then classified via ELM, and achieved 96.6% accuracy, whereas our proposed brain tumor classification approach attained the best accuracy of 99.7% and performed better than the existing methodologies.

The article "A Novel and Effective Brain Tumor Classification Model Using Deep Feature Fusion and Famous Machine Learning Classifiers" was published in 2022. Journal: Comput Intell Neurosci.

Table 8 compares the performance of the proposed feature fusion-based method with non-DL-based techniques. The authors in Thejaswini et al. [52] used the Adaptive Regularized Kernel-based Fuzzy C-Means Clustering (ARKFCM) approach to segment images and extract statistical features from the segmented area. Using the SVM, the system achieved a success rate of 91.4%. Kaplan et al. [53] suggested an approach that uses Local Binary Pattern (LBP) as a feature extraction technique and KNN as a classification technique. The system achieved the highest accuracy of 95.5%. Chen et al. [28] evaluated the effectiveness of various feature extraction methods such as density histogram, grey level cooccurrence matrix (GLCM), and Bag of Word (BoW). They attained the highest accuracy of 91.4% with SVM and KNN as classifiers and BoW as a feature extraction method. The traditional approaches usually rely on manual tumor segmentation and feature extraction, which is both time-consuming and error-prone. To find an optimal solution, these techniques need to be tried and tested by a knowledgeable expert.

CNNs have made significant advances in image processing, allowing any classification or segmentation operation to be performed precisely, crucial in biomedical applications. This research proposes a novel brain tumor classification technique based on the fusion of deep features extracted using three distinct CNN architectures. The proposed brain tumor classification framework is an efficient and segmentation-free approach that employs a hybrid feature set. The fusion of multiple feature vectors produces a more discriminative feature representation than an independent vector. Usually, the features extracted from different CNN architectures are more robust and descriptive than those obtained from homogenous CNN architectures or a single CNN architecture because of the diverse range of low-level and high-level features.

The dataset used in this study, however, is imbalanced. In general, a well-balanced data set with an equal class distribution yields better prediction accuracy. It is worth noting that a well-balanced dataset makes learning easier for the classification system. The dataset used in this study is available publicly; thus, the class imbalance is obvious. Hence, the dataset used in this study is extensively augmented to deal with the class imbalance problems. Moreover, due to the imbalanced dataset, the proposed framework is also assessed using recall, precision, and f1-score. The results prove that the proposed framework can be deployed in a clinical setup for real-time diagnosis of brain tumors.

The article "A Novel and Effective Brain Tumor Classification Model Using Deep Feature Fusion and Famous Machine Learning Classifiers" was published in 2022. Journal: Comput Intell Neurosci.

## 6. Conclusion and Future Work

This paper presents a novel deep feature fusion-based framework to classify brain tumors from MR images. The proposed framework extracts a wide range of low-level and high-level features from AlexNet, GoogLeNet, and ResNet18 architectures with varying depth and design. These features are then merged using a serial fusion approach to generate a single vector. The novel feature vector contains robust combination features classified using SVM and KNN. The proposed method is trained and evaluated on 15,320MR images and obtained accuracy of 99.7%, recall value of 1.0, a precision score of 0.99, and 0.99 *f*1-score. The novel feature vector outperformed the independent CNN feature vectors. Moreover, the feature fusion strategy aids in overcoming the drawbacks of a single CNN model, thus resulting in higher performance, particularly for larger datasets. The obtained results prove the efficacy and robustness of the proposed method in brain tumor classification. Hence, the proposed framework can assist radiologists in detecting and classifying brain tumors accurately. In the future, we will explore other CNNs such as VGG, DenseNet, and machine learning classifiers such as Random Forests and Ensemble learning. Moreover, additional MRI datasets will be gathered with other tumor categories and different imaging modalities for classification.

## Figures and Tables

**Figure 1:** Diagram illustrating the architecture of proposed method.

**Figure 2:** MRI before and after normalization.

**Figure 3:** Various image augmentation techniques applied on Figshare dataset. (a) Original image. (b) 45-degree rotation. (c) Right/left mirroring. (d) Upside down flip. (e) Salt/pepper noise.

**Figure 4:** General CNN architecture.

**Figure 5:** Modifying CNN architecture for application.

**Figure 6:** CNN architectures of (a) AlexNet, (b) ResNet18, and (c) GoogLeNet [17].

**Figure 7:** Serial based fusion of deep feature vectors.

**Figure 8:** Depiction of normalized MRIs at different planes.

**Figure 9:** Dataset distribution ratio.

**Figure 10:** Recall, precision, and *F*1-score values obtained from SVM and KNN.

**Figure 11:** Confusion matrix obtained from (a) SVM and (b) KNN.

**Figure 12:** ROC curves for (a) glioma, (b) meningioma, and (c) pituitary.

**Table 1:** Number of images before and after augmentation.

Tumor type	Images before augmentation	Images after augmentation
Pituitary	930	4650
Glioma	708	3540
Meningioma	1426	7130
Total	3064	15,320

The article "A Novel and Effective Brain Tumor Classification Model Using Deep Feature Fusion and Famous Machine Learning Classifiers" was published in 2022. Journal: Comput Intell Neurosci.

**Table 2:** Parameters of deep learning models.

CNN	Input size	Depth	Parameters (M)
GoogLeNet	224 × 224	22	7
ResNet18	224 × 224	18	11
AlexNet	227 × 227	8	61

**Table 3:** Total no. of MRI slices in each tumor type along with the number of patients.

Type of tumor	No. of patients	No. of images
Glioma	91	1426
Pituitary	60	930
Meningioma	82	708
Total	233	3064

**Table 4:** Training parameters for CNNs.

Hyper-parameters	Values
Epoch	30
Mini-batch size	10
Optimizer	SGDM
Learning rate	1*e* − 4

**Table 5:** Accuracy % obtained from independent and fused feature vectors.

Feature vector/Classifiers	Accuracy %	
	SVM	KNN
GoogLeNet	97.6	97.6
ResNet18	98.0	97.7
AlexNet	97.9	98.0
Fused	99.7	99.7

**Table 6:** Class-wise evaluation metrics obtained from confusion matrix.

Tumor type	*F*1-score	Recall	Precision
Glioma	1.0	1.0	1.0
Meningioma	0.99	1.0	0.99
Pituitary	1.0	1.0	1.0
Average	0.99	1.0	0.99

**Table 7:** Comparison of proposed techniques with the existing systems.

Reference	Technique	Accuracy%
Anarkari et al. [30]	CNN	94.2
Afshar et al. [32]	CapsNet	90.8
Sejuti and Islam [50]	CNN + SVM	97.1
Kang et al. [8]	DenseNet169 + Inception-v3 + ResNeXt50	98.5
Ari et al. [23]	AlexNet + VGG16	96.6
Proposed	AlexNet + GoogLeNet + ResNet18	99.7

**Table 8:** Comparison with traditional ML techniques.

Reference	Technique/s	Accuracy (%)
Chen et al. [51]	BoW, GLCM, SVM, and KNN	91.4
Thejaswini et al. [52]	ARKFCM and SVM	91.4
Kaplan et al. [53]	LBP and KNN	95.5
Proposed	CNN, SVM, and KNN	99.7

## Data Availability

The data used to support the findings of this study are available from the corresponding author upon request.
